The article "The effects and safety of pirfenidone in the treatment of idiopathic pulmonary fibrosis: a meta-analysis and systematic review" was published in 2021. Journal: Eur J Med Res.

# The effects and safety of pirfenidone in the treatment of idiopathic pulmonary fibrosis: a meta-analysis and systematic review

**DOI:** 10.1186/s40001-021-00601-y

**Published:** 2021-10-30

**Authors:** Chenchen Zang, Yan Zheng, Yanqing Wang, Lisha Li

**Affiliations:** 1 Department of Respiratory and Critical Care Medicine, Qingdao Hospital of Traditional Chinese Medicine(Qingdao Hiser Hospital), No.4 Renmin Road, Shibei District, Qingdao, 266000 Shandong Province China; 2 Department of General Practice, Qingdao Hospital of Traditional Chinese Medicine(Qingdao Hiser hospital), Qingdao, China

**Keywords:** Pirfenidone, Idiopathic pulmonary fibrosis, Effect, Safety, Treatment

## Abstract

**Background:**

It is necessary to systematically evaluate the efficacy and adverse reactions of pirfenidone in the treatment of patients with idiopathic pulmonary fibrosis (IPF).

**Methods:**

Pubmed et al. databases were searched up to March 15, 2021 for randomized controlled trials (RCT) of pirfenidone in the treatment of IPF. Two authors collected and compared the indicators including progression-free survival (PFS), vital capacity (VC), forced vital capacity (FVC), and adverse reactions. RevMan 5.3 software and Stata 15.0 software were used for meta-analysis.

**Results:**

A total of 8 reports with 9 RCTs involving 1824 IPF patients were included. Meta-analysis results showed that compared with the control group, pirfenidone could prolong the PFS phase of IPF patients (HR = 0.65, 95% CI 0.55 ~ 0.76, *P* < 0.001), slow down the VC of IPF patients (SMD = 0.43, 95% CI 0.21 ~ 0.66, *P* < 0.001), and decrease FVC (SMD = 0.31, 95% CI 0.14 ~ 0.48, *P* < 0.001). The main adverse reactions of pirfenidone were gastrointestinal reactions, photosensitivity and skin rashes.

**Conclusion:**

Pirfenidone is beneficial to prolong the PFS of IPF patients, improve lung function, and it is safe for clinical use. However, more high-quality RCTs are still needed to provide reliable evidence for the treatment of IPF.

## Background

Idiopathic pulmonary fibrosis (IPF) is a kind of unexplained, chronic progressive fibrotic interstitial pneumonia, and it is more likely to occur in middle-aged and elderly people [1]. The global annual incidence of IPF is 0.2 per 100,000 to 93.7 per 100,000, and it is increasing over time [2]. It has been reported that the annual incidence of IPF in Taiwan from 2000 to 2007 was 2.8 per 100,000 to 6.4 per 100,000, with the highest incidence in men over 75 years of age [3, 4]. Most patients have rapid disease progression and short survival time after being diagnosed with IPF [5]. Once fibrotic alterations occur, it is difficult to reverse, and early diagnosis and treatment are particularly important to the prognosis of IPF patients [6].

The article "The effects and safety of pirfenidone in the treatment of idiopathic pulmonary fibrosis: a meta-analysis and systematic review" was published in 2021. Journal: Eur J Med Res.

The previous treatment of IPF often included hormones and immunosuppressive agents, with the goal of reducing inflammation as much as possible and delaying the progression of inflammation to fibrosis [7, 8]. With the deepening of research, the pathogenesis has changed from “initiating factors of inflammation” to “fibrosis in the repair of alveolar epithelial injury”, and drug treatment has also gradually changed from "anti-inflammatory" to "anti-fibrosis", but there is still no drug that can completely cure IPF [9, 10]. New anti-fibrosis drugs seem to delay the progression of the disease and are recommended by domestic and foreign guidelines for the treatment of IPF [11]. Pirfenidone was approved for use in China in December 2013. In view of the current limited clinical application report data of pirfenidone and the inconsistent results of related studies for technical limitations of randomized controlled trials (RCTs), this present meta-analysis aimed to systematically evaluate the efficacy and safety of pirfenidone in the treatment of IPF, to provide evidence to the IPF treatment and clinical drug use.

## Methods

This meta-analysis and systematic review was conducted and reported in comply with the Preferred Reporting Items for Systematic Reviews and Meta-Analyses (PRISMA) [12].

### Search strategy

Two investigators conducted computer search of Cochrane Library, PubMed, EMBase, China national knowledge infrastructure (CNKI), Chinese Biomedical Literature Database and Wanfang Database for RCTs on the applications of pirfenidone in the treatment of IPF, the search time limit was from the establishment of each database to March 15, 2021. Following search terms were applied: "Pirfenidone"," idiopathic pulmonary fibrosis ", “IPF”, “pulmonary fibrosis”, “randomized controlled trial”, “RCT”.

### Inclusion and exclusion criteria

The inclusion criteria for RCTs in this meta-analysis were: ① RCT design on the pirfenidone use in the treatment of patients with IPF; ② all patients met the diagnostic criteria for IPF, and the experimental group was treated with pirfenidone and other clinical treatments were the same as the control group, the control group adopted conventional treatment methods using placebo or blank control, and the treatment duration was at least 3 months; ③ evaluation indicators were reported such as disease progression-free survival (PFS), vital capacity (VC), forced vital capacity (FVC), adverse reactions, etc.

The exclusion criteria in this meta-analyses were: ① duplicate publication; ② studies with failure to provide sufficient original data.

The article "The effects and safety of pirfenidone in the treatment of idiopathic pulmonary fibrosis: a meta-analysis and systematic review" was published in 2021. Journal: Eur J Med Res.

### Literature screening and data extraction

Two investigators independently screened and cross-checked the literature according to the inclusion and exclusion criteria. In case of disagreement, they discussed or consulted a third party to assist in the judgment. Then two authors extracted the following information independently according to the designed data extraction table: author, publication year, basic information of the research population, sample size, treatment plan, outcome indicators and related data. The original authors were contacted as much as possible for the lack of related outcome data.

### Quality evaluation

The Cochrane Collaborations risk of bias tool [13] was used to evaluate the methodological quality and risk of bias of included RCTs, any disagreements in the quality evaluation were resolved by discussion and consensus. The Cochrane risk of bias tool includes seven specific domains: sequence generation, allocation concealment, blinding of participants and personnel, blinding of outcome assessment, incomplete outcome data, selective outcome reporting and other issues. Every domain could be classified as low risk of bias, high risk of bias or unclear risk of bias according to the judgment criteria.

### Statistical analysis

RevMan 5.3 software and Stata 15.0 software were used for meta-analysis. Firstly, a heterogeneity test on the synthesized data was conducted. If *P* > 0. 1, *I*^2^ < 50%, it was considered as homogeneous among multiple studies, and a fixed effects model was used for meta-analysis; if *P* < 0. 1. If *I*^2^ ≥ 50%, it was considered that there was heterogeneity in the effect size, then the source of heterogeneity was analyzed by conducting subgroup analysis, sensitivity analysis and applied random effects model. The effect size of each study was calculated according to the method of Parmar et al., and the combined effect size, combined weight and 95% CI were calculated. Publication bias was evaluated by using funnel plots, and asymmetry was assessed by conducting Egger regression test. In this meta-analysis, the difference was statistically significant with *P* < 0.05.

## Results

### Study inclusion

As shown in Fig. 1, 104 related reports were retrieved for the first time. After reading the title and abstract, 68 studies were excluded. Based on the inclusion and exclusion criteria, the documents that did not meet the inclusion criteria were removed, and 8 reports [14–21] with 9 RCTs were finally included. The conditions of all reported cases were in a stable phase. The total number of patients was 1824, with 930 cases in the experimental group, and 894 cases in the control group. The basic information of the included studies is shown in Table 1.

The article "The effects and safety of pirfenidone in the treatment of idiopathic pulmonary fibrosis: a meta-analysis and systematic review" was published in 2021. Journal: Eur J Med Res.

**Fig. 1:** PRISMA flow diagram

**Table 1:** The characteristics of included RCTs

Study ID	Sample size			Interventions		Durations	Outcomes
	Experimental group	Control group		Experimental group	Control group		
Azuma 2005	72	35		Pirfenidone 1800 mg/d	Placebo	9 months	Pirfenidone is not yet able to increase the lowest SpO_2_ in 6MWT, but it can increase the VC of IPF patients
CAPACITY 004 2011	174	174		Pirfenidone 2403 mg/d	Placebo	72 weeks	Pirfenidone slowed the decline of FVC and prolonged the PFS period, but did not significantly increase the lowest SpO 2 of 6MWD and 6MWT
CAPACITY 006 2011	171	173		Pirfenidone 2403 mg/d	Placebo	72 weeks	Pirfenidone did not increase the lowest SpO 2 in FVC, PFS phase and 6MWT, but pirfenidone could reduce the decline of 6MWD
Huang 2015	38	38		Pirfenidone 1800 mg/d	Placebo	48 weeks	The pirfenidone group can significantly prolong the PFS period, without significantly delaying the decline of FVC, and not increasing the lowest SpO_2_ of 6MWD and 6MWT
King 2014 (ASCEND)	278	277		Pirfenidone 1800 mg/d	Placebo	52 weeks	Pirfenidone can slow down the decline of FVC and 6MWD, and significantly prolong the PFS
Lei 2018	20	20		Pirfenidone 1200 mg/d	Blank control	48 weeks	Pirfenidone can delay the decline of FVC
Li 2015	43	44		Pirfenidone 1200 mg/d	Placebo	48 weeks	Pirfenidone can improve FVC and slow down the decline of 6MWD
Li 2016	24	24		Pirfenidone 1200 ~ 1800 mg/d	Blank control	6 months	Pirfenidone can improve FVC and increase 6MWD
Taniguchi 2010	110	109		Pirfenidone 1800 mg/d	Placebo	52 weeks	Pirfenidone can slow down the decline of VC in IPF patients and prolong the PFS

*PFS* progression-free survival, *VC* vital capacity, *FVC* forced vital capacity

### Quality of included studies

We used the bias risk assessment tool recommended by Cochrane Network for quality evaluation. Among the 9 included RCTs, 7 of the included studies [14, 16–20] had clear randomization schemes, the patients were randomized according to the random number table method or computer randomization method. The randomization plan of two RCTs is not clear. 7 studies [14, 16, 17, 19–21] reported allocation concealments, and 5 RCTs [14, 17, 19, 20] reported the blinding design on the participants and personnel. All the included studies did not report the blinding design on the outcome assessment. No other significant biases in the incomplete outcome data, selective reporting and other biases were found (Figs. 2, 3).

**Fig. 2:** Risk of bias graph

**Fig. 3:** Risk of bias summary

### Synthesized outcomes

*PFS* 5 RCTs [15, 18–20] reported the effect of pirfenidone on PFS in patients with IPF. The results of meta-analysis showed that there was no heterogeneity among the studies (*I*^2^ = 0%, *P* = 0.525), and the fixed effects model was selected. Compared with control group, pirfenidone significantly prolonged the PFS of IPF patients (HR = 0.65, 95% CI 0.55 ~ 0.76, *P* < 001, Fig. 4).

The article "The effects and safety of pirfenidone in the treatment of idiopathic pulmonary fibrosis: a meta-analysis and systematic review" was published in 2021. Journal: Eur J Med Res.

**Fig. 4:** The plot forest of PFS

*VC* 2 studies [14, 20] reported the changes in VC of IPF patients. Meta-analysis results showed that there was no heterogeneity between studies (*I*^2^ = 0%, *P* = 0.818), and the fixed effects model was selected. Compared with control group, pirfenidone could slow down the decline of VC in IPF patients (SMD = 0.43, 95% CI 0.21 ~ 0.66, *P* < 0.001, Fig. 5).

**Fig. 5:** The plot forest of VC

*FVC* 6 studies [15–19] reported the change of FVC from the baseline value. The results of meta-analysis showed that there was heterogeneity among the studies (*I*^2^ = 72. 6%, *P* = 0.003), and the random effects model was selected. Compared with control group, pirfenidone could delay the decline of FVC in IPF patients (SMD = 0.31, 95% CI 0.14 ~ 0.48, *P* < 001, Fig. 6). Due to different follow-up times, some studies reported changes in FVC values at multiple time points. Meta-analysis showed that the reported studies had homogeneity (all *I*^2^ < 50%), and fixed-effect models were selected. Compared with the control group, at 48–52 weeks and 72 weeks, Pirfenidone slowed down the decline of FVC in IPF patients (SMD = 0.40, 95% CI 0.14 ~ 0.67, *P* = 0.003; SMD = 0.21, 95% CI 0.06 ~ 0.36, *P* = 0.006).

**Fig. 6:** The plot forest of FVC

*Adverse complications* The included reports had reported the adverse reactions of pirfenidone in the treatment of IPF, but there is a large heterogeneity among the studies (*I*^2^ = 88.15%, *P* < 0.001), because it is impossible to determine the source of heterogeneity, descriptive integration is used. As shown in Table 2, the incidence of adverse events in the two groups of patients was relatively high. Most of the adverse events were mild to moderate, and symptoms disappeared after dose reduction or discontinuation of pirfenidone and symptomatic treatment. In the studies of Azuma [14], CAPACITY [19], Huang^15^, and Lei [17], the differences in the results of the adverse reactions between the groups were statistically significant, while the results of the studies by Taniguchi^20^ and Li^21^ were not statistically significant. In several studies, there were no interruption of treatment due to serious adverse events, which might be related to the small sample size and the small oral dose.

**Table 2:** Adverse reactions of pirfenidone treatment

Study ID	Main adverse reactions	Major adverse reactions leading to interruption of treatment
Azuma 2005	Photosensitivity (43.8%), gastrointestinal discomfort (30.1%), anorexia (31.5%)	Photosensitivity (5 cases), vomiting, fever, abnormal liver function, dizziness, facial paralysis, hepatocellular tumor (1 case each)
CAPACITY 2011	Nausea (36.0%), skin rash (32.0%)	Nausea (36.0%), rash (28.1%), headache (25.9%), cough (25.2%), diarrhea (22.3%)
Huang 2015	Skin rash (39.5%), nausea (5.26%), diarrhea (7.89%)	NA
King 2014	Nausea (36.0%), rash (28.1%), headache (25.9%), cough (25.2%), diarrhea (22.3%)	Acute exacerbation of IPF, elevated liver enzymes, pneumonia (both 1.1%)
Lei 2018	Photosensitivity, loss of appetite, fatigue	NA
Li 2015	NA	NA
Li 2016	Gastrointestinal reaction, abnormal liver function	NA
Taniguchi 2010	Photosensitivity (51.4%), nasopharyngitis (49.5%), anorexia (16.5%)	Photosensitivity (2.8%), lung cancer (1.8%), fever (1.8%), respiratory failure (1.8%)

The article "The effects and safety of pirfenidone in the treatment of idiopathic pulmonary fibrosis: a meta-analysis and systematic review" was published in 2021. Journal: Eur J Med Res.

### Publications of bias

We attempted to evaluate publication bias by using a funnel plot if ten or more RCTs were included in outcome meta-analysis. Limited by the number of included RCTs, we could not perform funnel plot. Egger regression tests indicated that there was no significant publication of biases (all *P* > 0.05).

Sensitivity analyses, which investigate the influence of 1 study on the overall risk estimate by removing one study in each turn, suggested that the overall risk estimates were not substantially changed by any single study.

## Discussion

The pathogenesis of IPF is complex, and it is not yet fully clear. There are fewer effective drugs for the treatment of IPF in the clinic, so although the incidence of the disease is low, the prognosis is extremely poor [22, 23]. Several studies [24–26] have proved that pirfenidone has anti-fibrosis, anti-oxidation and anti-inflammatory effects. It mainly inhibits transforming growth factor (TGF)-β, tumor necrosis factor (TNF)-α and platelet-derived growth factor (PDGF) to produce an anti-fibrosis effect. Pirfenidone is a pleiotropic pyridine compound that reduces the extracellular matrix by inhibiting the synthesis of collagen stimulated by transforming growth factor β, and prevents the proliferation of fibroblasts to achieve anti-fibrosis, anti-inflammatory and anti-oxidant effects [27, 28]. It has been reported that antioxidant activity mediates pirfenidone antifibrotic effects in human pulmonary vascular smooth muscle cells exposed to sera of idiopathic pulmonary fibrosis patients [29]. Besides, pirfenidone exerts beneficial effects on specific markers of oxidative stress and inflammation in IPF patients [30]. The results of this meta-analysis have showed that compared with the control group, pirfenidone reduces the risk of IPF progression or death by 35%, and it can significantly improve lung function, including delay the decline of VC and FVC. Although almost all patients have different degrees of adverse reactions, mainly including gastrointestinal reactions such as nausea and diarrhea, photosensitivity and skin rashes, most of them are mild to moderate. After drug reduction, discontinuation and symptomatic treatment, the symptoms can disappear. Although serious adverse reactions such as tumors, abnormal liver function, and respiratory failure have occurred, they are rare. Therefore, pirfenidone can effectively improve the quality of life of IPF patients and is safe for clinical use.

The article "The effects and safety of pirfenidone in the treatment of idiopathic pulmonary fibrosis: a meta-analysis and systematic review" was published in 2021. Journal: Eur J Med Res.

A number of studies [31–33] have investigated the efficacy of bosentan, imatinib, etanercept, interferon gamma, and prednisone, azathioprine and N-beta cysteine in the treatment of IPF. However, the results of the related studies show that the efficacy of each drug in the treatment of IPF is unsatisfactory. Therefore, finding effective drugs for the treatment of IPF is always one of the hot spots in this research field. Pirfenidone is an anti-fibrosis drug with anti-fibrosis, anti-inflammatory and antioxidant effects [34, 35]. However, existing guidelines recommend pirfenidone for the treatment of mild and moderate IPF, but its mechanism of action is still unclear and needs to be further explored.

Studies [36] have reported that the overall incidence of adverse reactions during the use of pirfenidone in China post-marketing patients is 8.90%. Most of the adverse reactions that occurred are mild to moderate and can be tolerated. There was no discontinuation of treatment due to adverse reactions happened so far, there have been no reports of serious adverse events related to drugs. The most common adverse reactions of pirfenidone are gastrointestinal reactions, skin allergic reactions, and elevated transaminases [37]. The other common side effects of nintedanib, another IPF treatment drug, are diarrhea, elevated transaminases, bleeding, etc. The side effects of those two drugs have similar symptoms. Studies [38–40] have reported that patients who are older than 60 years old and whose dosage of pirfenidone is greater than 1.2 g/day have a high probability of adverse reactions. Therefore, patients should be cautious when using high-dose pirfenidone. Meanwhile, more clinical studies are needed to further explore the effectiveness and safety of different doses of pirfenidone in patients with IPF.

This meta-analysis has certain limitations. First of all, among the 8 included reports, most of the studies have scientific and rigorous experimental design, with high patient compliance, low loss to follow-up, and high quality. However, there are still several RCTs did not explained the specific random allocation methods and blinding design. The above factors are the main reasons for the high-risk bias, and it may be the important reasons for the large heterogeneity of the results. Additionally, the included RCTs did not report in detail whether pirfenidone can reduce the mortality of IPF patients. Therefore, more large samples and high-quality RCTs are needed to further confirm the efficacy and safety of pirfenidone on IPF.

The article "The effects and safety of pirfenidone in the treatment of idiopathic pulmonary fibrosis: a meta-analysis and systematic review" was published in 2021. Journal: Eur J Med Res.

## Conclusions

In summary, pirfenidone is beneficial for prolonging the PFS phase of patients with IPF, improve lung function with good safety. It is recommended for clinical IPF treatment, but clinicians still need to make a reasonable choice based on the patient's condition. With the development of medicine, it is still necessary to design larger sample size and more scientific RCTs to verify the therapeutic effect and safety of pirfenidone in patients with IPF, to provide more reliable medical evidence for the treatment of IPF.

## Data Availability

All data generated or analyzed during this study are included in this published article.

## Abbreviations

IPF: Idiopathic pulmonary fibrosis
RCT: Randomized controlled trials
PFS: Progression-free survival
VC: Vital capacity
FVC: Forced vital capacity
PRISMA: Preferred Reporting Items for Systematic Reviews and Meta-Analyses
CNKI: China national knowledge infrastructure
TGF: Transforming growth factor
TNF: Tumor necrosis factor
PDGF: Platelet-derived growth factor
